The article "The Effects of Fetal Gender on Serum Human Chorionic Gonadotropin and Testosterone in Normotensive and Preeclamptic Pregnancies" was retracted in 2013. Reasons: plagiarized text; overlap with other authors' work.

# The Effects of Fetal Gender on Serum Human Chorionic Gonadotropin and Testosterone in Normotensive and Preeclamptic Pregnancies

**DOI:** 10.1155/2012/874290

**Published:** 2012-02-15

**Authors:** Nahid Lorzadeh, Sirous Kazemirad

**Affiliations:** Department of Obstetrics and Gynecology, Asali Hospital, Lorestan University of Medical Sciences, Lorestan, Iran

## Abstract

*Introduction*. The aim of the present study was to evaluate the effects of fetal sex on serum human chorionic gonadotropin (hCG) and testosterone in normotensive and preeclamptic pregnancies. *Materials and Methods*. This is a cross-sectional study and 139 women with singleton pregnancies in the third trimester were studied. Seventy-one pregnancies were uncomplicated; among those were 35 male and 36 female fetuses. Sixty-eight pregnancies were complicated by preeclampsia; among those were 35 male and 33 female fetuses. Human chorionic gonadotropin and total testosterone were measured in maternal peripheral blood. Data analyzed by SPSS software. *Results*. In male-bearing pregnancies, maternal hCG and testosterone serum levels were significantly higher in preeclamptic than normotensive mothers (*P* < 0.001 and *P* < 0.001, resp.) in female-bearing pregnancies testosterone levels were significantly higher in preeclamptic than normotensive mothers (*P* < 0.001). Total testosterone levels were significantly higher in pregnancies with either gender and significantly higher in mlae-bearing than in female-bearing pregnancies. *Conclusion*. According to our results, there is a correlation between maternal serum hCG and testosterone levels and preeclampsia. Therefore these tests can be used as routine during 30–38 weeks of gestation. High maternal serum concentrations of these markers can predict preeclampsia.

## 1. Introduction

Following the inflammation cascade, placenta produces some peptides that might be valuable as predictive markers of preeclampsia. Some studied peptides in this field include corticotrophin-releasing hormone (CRH, hCG), human chorionic gonadotropin, activin A, and inhibin A. Since the disease is resolved soon after delivery, most attention is focused on fetus, placenta, and fetal membranes. hCG concentration in maternal blood is 100 U/L during miss period. At 8–10 weeks of gestation, hCG level rises to a peak of 100,000 U/L, then drops down to 10000–20000 U/L at 18–20 weeks and reaches a plateau for the rest of the pregnancy [1]. During the first and second trimesters of normal pregnancy, there are no gender differences in maternal hCG levels. However, from the second to the third trimesters, there is a marked shift in maternal hCG serum concentrations. The hCG levels in female-bearing pregnancies increase significantly, whereas they decrease in male-bearing pregnancies [1–3]. Maternal serum concentration of total testosterone (TT) increases gradually throughout pregnancy, whereas free testosterone (FT) levels change very little until the third trimester and then become double. The sources for the increased testosterone levels in maternal serum are unknown but could be the ovarian theca-interstitial cells and the maternal cortex, which might be stimulated by hCG throughout pregnancy [4].

The article "The Effects of Fetal Gender on Serum Human Chorionic Gonadotropin and Testosterone in Normotensive and Preeclamptic Pregnancies" was retracted in 2013. Reasons: plagiarized text; overlap with other authors' work.

Gurbuz et al. in a study in 2004 found that the maternal serum hCG level is a useful laboratory tool when managing and treating hypertensive disorders that complicate pregnancy [5]. An increased level of serum hCG is found in mothers with pregnancies complicated by preeclampsia. On the other hand, testosterone levels have been shown to be significantly higher in preeclamptic pregnancies than normal pregnancies [6–8]. Steier et al. in a study in 2002 found that in male-bearing pregnancies maternal serum hCG and testosterone levels are significantly higher in preeclamptic mothers than normotensive mothers [2, 9–11]. Gol et al. in 2004 found that hCG concentration in maternal serum and cord blood is significantly higher in normal pregnancies with female than male fetuses [3, 12]. Elsmén et al. concluded that mean serum hCG level in male-carrying pregnancies was significantly higher in preeclamptic pregnancies than in normal pregnancies [13]. Due to these limited data about the relationship between fetal gender and preeclampsia, this study was undertaken to investigate the effects of fetal gender on maternal serum concentration of hCG and testosterone in normotensive and preeclamptic pregnancies.

## 2. Materials and Methods

All pregnant women admitted to our outpatient obstetric clinic of Haj Asali Hospital for pregnancy visits from 23 October 2008 to 22 September 2009 were enrolled in this cross-sectional study. All women underwent routine pregnancy examinations, and if they had a blood pressure equal to or higher than 140/90 mmHg, urine analyses were requested to detect proteinuria. Women who had a proteinuria between trace to 2+ and without any signs and symptoms of severe preeclampsia were considered as mild-to-moderate preeclampsia. Pregnancies with severe preeclampsia did not enter the study. Pregnancies with gestational diabetes and fetal anomalies were also excluded from the study. Finally a total of 139 mothers met the criteria to enter the study.

Of the 139 women in the study, 68 were preeclamptic and 71 were normotensive. Among preeclamptic pregnancies were 35 male fetuses and 33 female fetuses. Of the 71 normal pregnancies, 35 were male bearing and 36 were female bearing. All pregnancies were at 30–38 weeks of gestation. The study was approved by the Ethical Institutional Committee of Lorestan University. Written informed consent was obtained from all participants. The including criteria was the patients who were primigravid, had third trimester pregnancy, BP = 140/90 mmHg, and proteinuria = 300 mg in a 24 h urine sample. Patients with renal diseases, chronic hypertension, renal and urinary infection, fetal disorders, multiple pregnancy, and immunologic diseases were excluded from the study. Pregnant women without the above criteria were considered as control group. A questionnaire was completed for each patient including patient's age, gestational age, parity, the history of hypertension, diabetes mellitus, hypertension in family, diabetes mellitus in family, and tobacco consumption. After taking informed consents from all pregnant women who entered the study, they were examined physically. Blood pressure and urine specimens were collected, and detailed ultrasonographic structural examinations of the fetuses were performed. Simultaneously, blood samples were drawn from an antecubital maternal vein prior to delivery at the time of admission (30–38 wk of gestation) for examination of hCG and total testosterone. A total of 10 CC peripheral venous blood was taken from each woman and sent to the central laboratory of Asali Hospital. Venous blood was collected by venepuncture in 10 mL silicone-coated Vacutainer blood-collecting tubes containing no additives between 7:00 AM and 9:00 AM in a fasting state. Blood was allowed to clot at room temperature and was then centrifuged for 20 minutes at 2000 g. Aliquots of the serum were then stored at −20°C until they were required for the assay.

The article "The Effects of Fetal Gender on Serum Human Chorionic Gonadotropin and Testosterone in Normotensive and Preeclamptic Pregnancies" was retracted in 2013. Reasons: plagiarized text; overlap with other authors' work.

Consistent with the definition of the ACOG, preeclampsia was defined as new-onset hypertension after 20 weeks of gestation, with a diastolic blood pressure of 90 mmHg or higher with concurrent proteinuria of 300 mg/24 hours or greater. Semiquantitative dipstick tests were used for measurement of proteinuria (1+ and 2+ corresponded to 300 mg/24 hours and 500 mg/24 hours, resp.). 10 human chorionic gonadotropin were measured by immunoradiometric assay (hCG IRMA KIT, IMMUNOTEC as Radova Prague). The Third International Standard for hCG was used as a reference standard. The assay has a detection limit of 3 IU/L. The intra-assay coefficient of variation was 3.3 and 7.0 for mean hCG levels at 21 and 1500 IU/L, respectively. The interassay coefficient of variation was 7.2 and 9.1 for hCG levels at 21 and 1500 IU/L, respectively.

Testosterone level was determined by a DRG Testosterone Eliza Kit (DRG Instruments GmbH, Germany). The test is based on a radioimmunoassay technique. The expected serum testosterone levels ranged between 0.3 and 2.8 nmol/L. The sensitivity was 0.1 nmol/L. The intra-assay coefficient of variation was 7.5 and 5.5 for testosterone levels at 1.6 and 26.5 nmol/L, respectively. The interassay coefficient of variation was 7.0 and 4.8 for testosterone levels at 1.2 and 23.3 nmol/L, respectively.

### 2.1. Statistical analysis

Laboratory tests results and other data (such as maternal age, gestational age, parity, type of pregnancy, systolic blood pressure, and diastolic blood pressure) were gathered in a questionnaire. Statistical analyses were performed using *t*-test and unparametric tests as appropriate, with statistical significance considered at *P* < 0.05. Data are presented as mean with standard error and 95% confidence interval (CI). SPSS version 15 was used to analyze the data.

## 3. Results

A total of 139 women with singleton pregnancies at 30–38 weeks of gestation entered the study. Maternal age was 14–38 years old, and parity was 0–3. In preeclamptic group, diastolic blood pressure was 90–110 mmHg and systolic blood pressure was 140–155 mmHg, and no difference was found between male and female fetuses (Table 1). Proteinuria was determined between +1 and +2, and it was not different between male and female fetuses. Mean serum hCG level was  16337 ± 2462 U/L in male-bearing normal pregnancies and  28774 ± 3197 U/L in female-bearing normal pregnancies. A statistically significant difference was found between the two mean values using *t*-test (*P* < 0.005). Mean serum hCG level was  31610 ± 3825 U/L in male-bearing preeclamptic pregnancies and 34480 ± 4559 U/L in female- bearing preeclamptic pregnancies. No significant difference was found between the two mean values using *t*-test (NS) (Table 2). Mean serum testosterone level in normal pregnancies was 2.85 ± 0.33 nmol/L for male fetuses and 2.50 ± 0.25 nmol/L for female fetuses. *t*-test showed no significant difference between the two mean values (NS). In pregnancies complicated with preeclampsia, mean serum testosterone level was 5.86 ± 0.78 nmol/L in male-carrying pregnancies and 3.92 ± 0.40 nmol/L in female-carrying pregnancies. The difference between mean values was statistically significant using *t*-test (*P* < 0.001) (Table 3). Mean serum hCG level in male-bearing pregnancies was significantly higher in preeclamptic (16337 ± 2462 U/L) than in normotensive pregnancies (31610 ± 3825) (*P* < 0.001) (Table 2). Mean serum hCG level in female-bearing pregnancies was not significantly different between normotensive (28774 ± 3197 U/L) and preeclamptic (34480 ± 4559 U/L) groups. Mean serum testosterone level in male-bearing pregnancies was significantly higher in preeclamptic group (2.85 ± 0.33 nmol/L) than in normotensive group (5.86 ± 0.78 nmol/L) (*P* < 0.001). Mean serum testosterone level in normotensive pregnancies with male fetus (2.50 ± 0.25 nmol/L) was found to be significantly lower than in female-bearing pregnancies complicated with preeclampsia (3.92 ± 0.40 nmol/L) (*P* < 0.001) (Table 3). Mean hCG serum level without considering fetus gender was shown to be  22643 ± 776 U/L in normal pregnancies and  33003 ± 339 U/L in preeclamptic pregnancies. The difference was shown significant using *t*-test (*P* < 0.001) (Table 4). Mean serum testosterone level without considering fetus sex was reported 2.67 ± 0.03 nmol/L in normal pregnancies and 4.92 ± 0.12 nmol/L for preeclamptic pregnancies (Table 5).

The article "The Effects of Fetal Gender on Serum Human Chorionic Gonadotropin and Testosterone in Normotensive and Preeclamptic Pregnancies" was retracted in 2013. Reasons: plagiarized text; overlap with other authors' work.

## 4. Discussion

These results are consistent with previous studies which also indicated that there is no gender difference in maternal serum hCG level during the first and second trimesters of pregnancy, but there is a shift from second to third trimester so that hCG levels significantly increase in female-bearing pregnancies and decrease in male-bearing pregnancies [9]. In a study by the American Association of Obstetricians and Gynecologists, it was reported that, in normal pregnancies, maternal serum hCG level is significantly higher in female-bearing pregnancies than in male-bearing pregnancies [12]. Several studies have found elevated hCG concentrations in maternal blood in preeclamptic pregnancies but without regard to fetal gender. Gurbuz et al. in a study in 2004 found that the maternal serum hCG level is a useful laboratory tool when managing and treating hypertensive disorders that complicate pregnancy. The serum hCG level is especially significant in severe preeclampsia and superimposed preeclampsia. Therefore, a high serum hCG level can be a helpful marker in the diagnosis and clinical management by preventing possible complications resulting from severe and superimposed preeclampsia [5]. In a study in Iran from 2001 to 2005, Basirat et al. found that maternal serum hCG level was significantly higher in preeclamptic pregnancies in comparison with normal pregnancies (*P* = 0.031) [6]. Bartha et al. in 2003 also indicated increased levels of maternal serum hCG in preeclamptic compared to normal pregnancies [14]. In the present study, the hCG levels in maternal blood in male-bearing preeclamptic pregnancies were significantly higher compared with that in male-bearing uncomplicated pregnancies, whereas in preeclampsia with female fetuses no significant increase in the maternal hCG level was observed. In a study in Turkey (2005), it was found that maternal serum hCG level at 24–28 weeks and 32–36 weeks of gestation is significantly higher in female-carrying pregnancies than male-bearing pregnancies (*P* < 0.004 and *P* < 0.001, resp.) [12]. Steier et al. in a study in 2002 found that in male-bearing pregnancies maternal serum hCG and testosterone levels are significantly higher in preeclamptic mothers than in normotensive mothers (*P* < 0.001). In female-bearing pregnancies, testosterone level was significantly higher in preeclamptic than normotensive mothers whereas hCG levels were not significantly different. Maternal serum levels of testosterone were significantly higher in preeclamptic pregnancies with male fetuses than with female fetuses (*P* < 0.001), whereas hCG levels were not significantly different. In normal pregnancies, female-bearing pregnancies had significantly higher serum hCG levels than male-bearing pregnancies (*P* < 0.005), whereas testosterone levels were not significantly different [9]. Elsmén et al. concluded that mean serum hCG level in male-carrying pregnancies was significantly higher in preeclamptic pregnancies than in normal pregnancies [13]. This finding was consistent with the study in America in which serum hCG level was found to be significantly higher in male-bearing pregnancies complicated with preeclampsia than normal ones (*P* < 0.001).

The article "The Effects of Fetal Gender on Serum Human Chorionic Gonadotropin and Testosterone in Normotensive and Preeclamptic Pregnancies" was retracted in 2013. Reasons: plagiarized text; overlap with other authors' work.

In the present study, mean serum hCG level was not significantly different between normal and preeclamptic pregnancies with female fetuses which was inconsistent with the results of the American Association of Obstetricians and Gynecologists. In fact, high maternal serum concentration of hCG in female-bearing pregnancies is not indicative of preeclampsia since this increment is also seen in normal pregnancies, whereas, in male-carrying pregnancies, high maternal serum levels of hCG can be a marker to predict preeclampsia. Mean serum hCG level was not significantly different in preeclamptic pregnancies with male and female fetuses which was in consistence with Steier et al.'s findings. Since there is an increment in maternal serum hCG levels in preeclamptic pregnancies with both male and female fetuses, so the difference between them is not clinically valuable. This finding suggested that the placenta seems to play a fundamental role in preeclampsia, as the condition improves rapidly after its removal. Examination of the placenta in pregnancies complicated by preeclampsia has revealed focal cellular necrosis with increased mitotic activity in the syncytiotrophoblast and cellular proliferation in the cytotrophoblast. A transformation of the cytotrophoblast into the syncytiotrophoblast also has been reported [15, 16].

The article "The Effects of Fetal Gender on Serum Human Chorionic Gonadotropin and Testosterone in Normotensive and Preeclamptic Pregnancies" was retracted in 2013. Reasons: plagiarized text; overlap with other authors' work.

These changes might explain the elevated maternal serum hCG levels in male-bearing preeclamptic pregnancies, but there is still no explanation for no increase in maternal serum hCG levels in female bearing with preeclampsia. In fact, high maternal serum concentration of hCG in female-bearing pregnancies is not indicative of preeclampsia since this increment is also seen in normal pregnancies, whereas, in male-carrying pregnancies, high maternal serum levels of hCG can be a marker to predict preeclampsia.

The serum levels of total testosterone increase throughout normal pregnancy and are primarily a result of progressive estrogen-induced increase in the concentration in sex-hormone-binding globulin concentrations [17, 18]. In preeclamptic pregnancies, however, studies have found lower maternal serum levels of estrogen than in normal pregnancies, so it is likely that other mechanisms mediate the maternal serum levels [19, 20]. In the present study, the maternal serum levels of total testosterone were significantly higher in preeclamptic than in normotensive pregnancies with male as well as with female fetuses (*P* < 0.001). Male-bearing preeclamptic pregnancies had significantly higher maternal serum testosterone levels than female-bearing pregnancies complicated by preeclampsia (*P* < 0.001).

The sources for the increased testosterone levels in maternal serum are unknown but could be the ovarian theca-interstitial cells and the maternal cortex, which might be stimulated by hCG throughout pregnancy. The fetal serum levels of testosterone are much lower than the maternal levels. Because of the stimulating effect of hCG on the fetal testis, the testosterone levels in male fetuses are significantly higher than in female fetuses. The fetal ovaries are regarded as hormone-ally inactive in the first part of pregnancy, but later they might have steroidogenic capacity [21–23].

In the present study, no correlations were found between maternal serum levels of hCG and total testosterone. In uncomplicated pregnancies, no significant gender differences were found. The significant increase in maternal serum testosterone levels in preeclamptic pregnancies with male fetuses as well as with female fetuses, and the significantly higher total testosterone maternal serum levels in male- than in female-bearing preeclamptic pregnancies were not related to maternal hCG levels only. In a study in 2006 in Athens, it was found that serum concentrations of total and free testosterone in preeclamptic pregnancies are significantly higher than in normal pregnancies (*P* < 0.01) [17]. Some other studies by Carlsen et al., Jirecek et al., and Gerulewicz et al. also showed increased levels of androgens in preeclamptic pregnancies in comparison with normal pregnancies [18–20]. It has been postulated that preeclampsia could result from a mutation in a paternally imprinted, maternally active gene. It is also known that only the paternal allele is expressed in human placenta [24, 25]. A paternal immunogenetic factor has been suggested, because significantly more preeclampsia is found in pregnancies with changed paternity [2, 26].

The article "The Effects of Fetal Gender on Serum Human Chorionic Gonadotropin and Testosterone in Normotensive and Preeclamptic Pregnancies" was retracted in 2013. Reasons: plagiarized text; overlap with other authors' work.

## 5. Conclusion

Our findings suggest the presence of an androgenic-mediated influence in the mechanism of preeclampsia. Considering high prevalence of preeclampsia and its complications on mother and fetus, most attempts are focused on prediction of the disease using detective indices. According to our results, there is a correlation between maternal serum hCG and testosterone levels and preeclampsia. Therefore, these tests can be used as routine during 30–38 weeks of gestation. High maternal serum concentrations of these markers can predict preeclampsia.

## Figures and Tables

**Table 1:** Comparison of the clinical characteristics in normal and preeclamptic pregnancies with male and female fetuses.

Type of pregnancy		Normal		Preeclamptic	
Fetal gender		Male	Female	Male	Female
Maternal age (year)	Range	14–38	17–28	14–39	15–36
	Mean ± SEM*	22.9 ± 0.9	21.2 ± 0.5	22.7 ± 1.2	22.5 ± 0.9
Parity (*n*)	Range	0–3	0–2	0–3	0–3
	Mean ± SEM	0.9 ± 0.2	0.6 ± 0.1	0.5 ± 0.1	0.5 ± 0.1
Gestational age (wk)	Range	30–37	31–37	30–38	30–37
	Mean ± SEM	33.5 ± 0.4	33.9 ± 0.3	34.1 ± 0.4	33.7 ± 0.4
Systolic blood pressure (mmHg)	Range	100–130	95–130	140–155	140–155
	Mean ± SEM	115.9 ± 1.6	113.5 ± 1.4	144.9 ± 0.8	145.5 ± 0.8
Diastolic blood pressure (mmHg)	Range	65–85	60–85	90–100	90–100
	Mean ± SEM	72.6 ± 1.2	70.6 ± 1.1	92.7 ± 0.5	92.9 ± 0.5

*SEM: standard error of the mean.

**Table 2:** Comparison of mean serum hCG level in normal and preeclamptic pregnancies with male and female fetuses.

Type of pregnancy	Normal		Preeclamptic		*P* value
Fetal gender	Number	hCG (mean ± SEM)	Number	hCG (mean ± SEM)	
Male	35	16337 ± 313	35	31610 ± 355	<0.001
Female	36	28774 ± 326	33	34480 ± 470	NS
*P* value		<0.005		NS	

**Table 3:** Comparison of mean serum testosterone level in normal and preeclamptic pregnancies with male and female fetuses.

Type of pregnancy	Normal		Preeclamptic		*P* value
Fetal gender	Number	Tes. (mean ± SEM)	Number	Tes. (mean ± SEM)	
Male	35	2.85 ± 0.03	35	5.86 ± 0.05	<0.001
Female	36	2.50 ± 0.02	33	3.92 ± 0.03	<0.001
*P* value		NS		<0.001	

**Table 4:** Comparison of mean serum hCG level between normal and preeclamptic pregnancies.

Type of pregnancy	Number	hCG (mean ± SEM)	*P* value
Normal	71	22643 ± 776	<0.001
Preeclamptic	68	33003 ± 339	
Total	139	27711 ± 614	

The article "The Effects of Fetal Gender on Serum Human Chorionic Gonadotropin and Testosterone in Normotensive and Preeclamptic Pregnancies" was retracted in 2013. Reasons: plagiarized text; overlap with other authors' work.

**Table 5:** Comparison of mean serum testosterone level between normal and preeclamptic pregnancies.

Type of pregnancy	Number	Testosterone (mean ± SEM)	*P* value
Normal	71	2.67 ± 0.03	
Preeclamptic	68	4.92 ± 0.12	<0.001
Total	139	3.77 ± 0.11	
